# The Effect of Probiotics in Stroke Treatment

**DOI:** 10.1155/2021/4877311

**Published:** 2021-10-28

**Authors:** Da-Yuan Zhong, Lan Li, Ruo-Meng Ma, Yi-Hui Deng

**Affiliations:** ^1^Guangdong Provincial Hospital of Integrated Traditional Chinese and Western Medicine, Foshan528200, China; ^2^HuNan University of Chinese Medicine, Changsha 410208, China

## Abstract

**Objective:**

We conducted a systematic review and meta-analysis to evaluate the curative effect of probiotics combined with enteral nutrition (EN) in patients with stroke.

**Methods:**

We retrieved randomized controlled trials and case-controlled trials on the use of probiotics for stroke treatment from PubMed, Web of Science, CNKI, Wanfang, and Weipu databases. Retrieval times were from the databases' inception to November 6, 2020. Two researchers conducted a strict evaluation of the literature quality and extracted the data, which were then entered into RevMan 5.3 for meta-analysis.

**Results:**

Twenty-three articles were included, including 1,816 patients. The meta-analysis revealed that probiotics combined with EN did not reduce NIHSS scores of patients with stroke (*P* > 0.05). However, it did shorten hospital stays and bedrest periods (*P* < 0.05). Probiotics combined with EN also improved patients' nutritional status and increased hemoglobin, albumin, serum total protein, and physical and chemical properties of prealbumin (*P* < 0.05). In terms of relieving inflammation, we found that probiotics combined with EN reduced neither high-sensitivity C-reactive protein nor procalcitonin (*P* > 0.05). However, it did cause a significant reduction in TNF-*α*, IL-6, and IL-10. Probiotics combined with EN significantly reduced esophageal reflux, bloating, constipation, diarrhea, gastric retention, and gastrointestinal bleeding. It relieved intestinal stress and reduced the occurrence of adverse reactions such as esophageal reflux, bloating, constipation, diarrhea, gastric retention, and gastrointestinal bleeding (*P* < 0.05). In terms of reducing stroke complications, probiotics combined with EN reduced the incidence of lung, gastrointestinal, and urinary tract infections (*P* < 0.05). It also reduced fatality rates and intestinal flora imbalance rates (*P* < 0.05).

**Conclusion:**

The probiotics combined with EN group's therapeutic effects were superior to those of the EN alone. Thus, probiotics combined with EN is worthy of both clinical application and promotion in stroke treatment.

## 1. Introduction

According to the latest World Health Organization report, stroke is the second leading cause of death worldwide [1]. In 2016 alone, around 5.5 million people died of stroke [2]. China has one of the world's heaviest stroke burdens; according to the latest census, the incidence of stroke in China is about 1.6% [3]. Damage to nerve function due to stroke affects gastrointestinal hormone and neurotransmitter secretion. In turn, this affects intestinal mucosa function, which leads to obstacles in the digestion and absorption of intestinal nutrients. Therefore, to ensure the body's nutritional supply, it is necessary to implant a nasogastric tube for enteral nutrition (EN). At present, the clinical nutritional support treatment consists primarily of parenteral nutrition and EN [4, 5]. However, long-term use of parenteral nutrition [6] may cause adverse reactions, such as catheter complications and intestinal mucosal injury. Additionally, EN promotes the proliferation of intestinal mucosal cells and maintains the gastrointestinal barrier function. Therefore, there is a low incidence of adverse reactions to EN. However, due to severe gastrointestinal dysfunction, patients with severe stroke are prone to complications such as diarrhea, constipation, and infection within 1 to 2 weeks after receiving EN support. This inhibits both the implementation and the effect of EN [7]. Probiotics are active microorganisms that are beneficial to the host and can form colonies in the human intestine. A balanced gut microecology has a positive and healthy effect on the human body. Wong [8] found that timely supplementation of probiotics can reduce intestinal permeability in critically ill patients, reduce pathogenic toxins and gas production, reduce abdominal distension, neutralize food allergies, reduce irritable bowel symptoms, and improve EN tolerance. As such, if a suitable entry point can be located, probiotics can be an effective treatment. Several clinical studies have confirmed the positive effects of probiotics in patients with stroke. However, due to the varying quality and sample sizes of these studies, there is no systematic means to evaluate the effects and safety of probiotic treatment combined with EN. Therefore, in this meta-analysis, we have consolidated published literature and provided a systematic review of evidence for the application of probiotics in patients with stroke.

## 2. Materials and Methods

### 2.1. Inclusion Criteria

#### 2.1.1. Study Types

Only clinical randomized controlled trials (RCTs) and case-controlled trials (CCTs) of probiotics for the treatment of stroke were included. We only included literature published in Chinese or English.

#### 2.1.2. Research Objects

The research subjects were patients with general clinical signs and symptoms of stroke (including ischemic stroke and hemorrhagic stroke) and without other diseases [9].

#### 2.1.3. Intervention Measures

We defined the treatment group as patients treated with probiotics combined with EN and life support treatment, and the control group as patients who received EN and life support treatment. There was no significant difference in either EN or life support between the two groups (*P* > 0.05).

#### 2.1.4. Outcome Indicators

First, we extracted the national institutes of health stroke scale (NIHSS) scores, average hospitalization time, average bedrest duration, time to reach the target supply of nutrient solution, hemoglobin (Hb), albumin (ALB), serum total protein (TP), physical and chemical properties of prealbumin (PA), tumor necrosis factor-*α* (TNF-*α*), high-sensitivity C-reactive protein (hs-CRP), procalcitonin (PCT), and interleukin-10 (IL-10) before and after treatment. Then, we extracted the incidence of adverse reaction indicators, such as vomiting, esophageal reflux, abdominal distension, constipation, diarrhea, gastric retention, and gastrointestinal bleeding. Then, we extracted the incidence of the three following complications: lung infection, gastrointestinal infection, and urinary tract infection. We also extracted the incidence of poor prognostic indicators, such as case fatality rate and flora imbalance. The calculation method [10] for the change of the mean value and the standard deviation was as follows, where *R* was the constant 0.5:

(1) $$\begin{array}{c} \text{mean}\left(\text{change}\right)=\text{mean}\left(\text{Before}\right)\text{mean}\left(\text{After}\right),\\ \text{sd}\left(\text{change}\right)=\sqrt{\text{sd}{\left(\text{Before}\right)}^{2}+\text{sd}{\left(\text{After}\right)}^{2}-2*R*\text{sd}\left(\text{Before}\right)*\text{sd}\left(\text{After}\right)}. \end{array}$$

### 2.2. Exclusion Criteria

Papers with inconsistent document types, documents with inconsistent intervention measures, duplicate documents, and documents without the above 24 outcome indicators were excluded.

### 2.3. Search Methods and Strategies

The databases searched were as follows: PubMed (https://pubmed.ncbi.nlm.nih.gov/), Web of Science (https://webofscience.com), China Knowledge Network (https://www.cnki.net/), Wanfang (Wanfangdata.com.cn/index.html), and Weipu (https://www.cqvip.com/). The search terms were as follows: stroke, cerebral infarction, ischemic stroke, hemorrhagic stroke, and probiotics. The retrieval time limit was from the databases' inception to November 6, 2020. The search strategy was as follows: we went through the search terms with free words and subject terms. Two researchers (Lan Li and Ruo-meng Ma) completed the retrieval operation. The search formula for PubMed was as follows:

  #7 Search: ((((stroke) OR (cerebral infarction)) OR (ischemic stroke)) OR (hemorrhagic stroke)) AND (probiotics)
  #6 Search: (((stroke) OR (cerebral infarction)) OR (ischemic stroke)) OR (hemorrhagic stroke)
  #5 Search: probiotics
  #4 Search: hemorrhagic stroke
  #3 Search: ischemic stroke
  #2 Search: cerebral infarction
  #1 Search: stroke

### 2.4. Data Extraction and Quality Evaluation

We entered the papers retrieved from each database into CNKI E-study to eliminate duplicates. According to the Patient, Intervention, Comparison and Outcome (PICO) principle, we read the titles and conducted an initial abstract screening. Then, we read the full texts and decided whether to include them in the study. For the RCT quality evaluation, we referred to the Cochrane risk bias assessment tool, which includes the following 7 evaluation items: random allocation method, allocation plan hiding, participant blinding, analyst blinding, resulting data completeness, selective reporting, and other biases. For the CCT quality evaluation, we referred to the Newcastle-Ottawa Scale, which includes the following 8 evaluation items: case definition adequacy, representativeness of the cases, selection of controls, definition of controls, comparability of cases and controls, and exposure ascertainment, which is the same method used to determine case and control exposure factors and nonresponse rate. Two of the authors (Da-yuan Zhong and Lan Li) completed quality evaluation of the studies. In the case of disagreement, the decision was made by a third author (Yi-hui Deng).

### 2.5. Statistical Analysis

We used RevMan5.3 for data analysis. Odds ratios (OR) and relative risk (RR) served as effect indicators for binary variables, and the weighted mean difference (MD) served as effect indicators for continuous variables. We used *t*^2^ and Chi^2^ statistics to analyze the heterogeneity between the studies. If *I*^2^ ≤ 50%, this indicated that the heterogeneity between the studies was minimal, and as such we used a fixed effects model. On the contrary, if heterogeneity was high, we used a random effects model. If there was greater heterogeneity between studies, we used subgroup analysis or sensitivity analysis. If there were few studies and high heterogeneity, we only performed a descriptive analysis.

## 3. Results

### 3.1. Retrieval Results and Basic Characteristics of the Included Studies

A total of 21 RCT articles and 2 CCT articles meeting the criteria were included in the sample [11–33], which included 1,816 patients. See Figure 1 for a flowchart of the literature search and inclusion flow and Table 1 for the basic characteristics of the included studies.

### 3.2. Evaluating Methodological Quality

We evaluated a total of 21 RCTs [11, 20, 22, 28, 30–33]. Eleven studies [11, 14, 20, 22, 24, 27, 28, 30, 31] mentioned specific randomization methods. None of the included studies mentioned allocation concealment methods or blinding methods. With the exception of 7 studies [11, 13, 15, 23, 25, 33], all studies had complete data. None of the studies had selective reporting. It is unclear whether there were other biases. As shown in Table 2, we assessed 2 CCTs [21, 29] for quality using the Newcastle-Ottawa Scale. All studies specified that the observation group and control group were taken from the same population. All studies mentioned that the baseline data for the two groups were comparable. This is shown in Table 3.

### 3.3. Meta-Analysis Results

#### 3.3.1. Effect on Stroke

The effect on stroke was assessed using the three following indicators: NIHSS score, hospital stay duration, and bed rest duration. The meta-analysis results showed that probiotics combined with EN did not significantly reduce the NIHSS scores (MD = -1.11, 95% confidence interval [CI] (−7.92, 5.70), *P*=0.75), but did significantly shorten hospitalization stay (MD = 8.94, 95% CI (−11.39, −6.50), *P* < 0.000001) and bed rest duration (MD = −10.34, 95% CI (−11.30, −9.39), *P* < 0.00001). These results are shown in Table 4.

#### 3.3.2. Blood Nutrition Indicators

The four blood nutrition indicators were HB, ALB, TP, and PA. The meta-analysis results showed that probiotics combined with EN increased HB (MD = 8.36, 95% CI (6.34, 10.38), *P* < 0.00001), ALB (MD = 2.91, 95% CI (2.45, 3.37), *P* < 0.00001), TP (MD = 4.90, 95% CI (2.43, 7.38), *P*=0.0001), and PA (MD = 15.50, 95% CI (9.2, 21.79), *P* < 0.00001) levels. These results are shown in Table 4.

#### 3.3.3. Inflammation Indicators

The five inflammation indicators were TNF-*α*, hs-CRP, PCT, IL-6, and IL-10. The meta-analysis results showed that probiotics combined with EN reduced TNF-*α* (MD = -3.22, 95% CI (−5.61,−0.82), *P* < 0.00001), IL-6 (MD = -16.40, 95% CI (−21.97, −10.83), *P* < 0.00001), and IL-10 (MD = −6.63, 95% CI (−12.55, −0.70), *P*=0.03) levels. However, it did not reduce hs-CRP levels (MD = −2.82, 95% CI (−10.10, 4.47), *P*=0.45) or PCT (MD = −0.35, 95% CI (−2.58, 1.89), *P*=0.76). These results are shown in Table 4.

#### 3.3.4. Adverse Reactions

Adverse events were assessed using 8 indicators: vomiting, esophageal reflux, abdominal distension, stress ulcer, constipation, diarrhea, gastric retention, and gastrointestinal bleeding. The meta-analysis results showed that probiotics combined with EN did not reduce the occurrence of vomiting (RR = 0.83, 95% CI (0.46, 1.51), *P*=0.55) or stress ulcers (RR = 0.47, 95% CI (0.22, 1.02), *P*=0.06). However, it did reduce esophageal reflux (RR = 0.43, 95% CI (0.25, 0.74), *P*=0.002) and bloating (RR = 0.39, 95% CI (0.26, 0.58), *P* < 0.00001), constipation (RR = 0.31, 95% CI (0.21, 0.45), *P* < 0.00001), diarrhea (RR = 0.22, 95% CI (0.14, 0.34), *P* < 0.00001), gastric retention (RR = 0.34, 95% CI (0.19,0.60), *P*=0.0002), and gastrointestinal bleeding (RR = 0.39, 95% CI (0.28, 0.54), *P* < 0.00001). These results are shown in Table 5.

#### 3.3.5. Complication Rate

Complications were assessed using the three following indicators: the incidence of lung infection, gastrointestinal infection, and urinary tract infection. The meta-analysis results showed that probiotics combined with EN reduced lung infection (RR = 0.44, 95% CI (0.27, 0.72), *P*=0.001), gastrointestinal infection (RR = 0.40, 95% CI (0.23, 0.68), *P*=0.0008), and urinary tract infection (RR = 0.27, 95% CI (0.15, 0.49), *P* < 0.0001), as shown in Table 5.

#### 3.3.6. Poor Prognostic Indicators

The poor prognostic indicators included the two following items: fatality rate and the intestinal flora imbalance rate. The meta-analysis results showed that probiotics combined with EN reduced the mortality rate (RR = 0.45, 95% CI (0.22, 0.93), *P*=0.03) and the bacterial imbalance rate (RR = 0.32, 95% CI (0.21, 0.48), *P* < 0.0001), as shown in Table 5.

#### 3.3.7. Publication Bias Analysis Results

We used a funnel chart to evaluate publication bias for adverse reactions, including bloating, constipation, diarrhea, and gastrointestinal bleeding. The funnel plots for bloating, constipation, and diarrhea had good symmetry, which suggests that there was a low possibility of publication bias in comparing these indicators. However, the diarrhea funnel chart had poor symmetry, which suggests that there may have been publication bias. The results of Egger's test were consistent with the results of the funnel chart, as shown in Figure 2.

## 4. Discussion

Stroke is an acute cerebrovascular disease that manifests primarily as blood vessel blockage in the brain. Stroke usually manifests as either ischemic or hemorrhagic and mostly occurs in men over 40 years old. The most common clinical treatments for stroke are drug therapy and thrombolytic therapy. Both of these treatments have a high risk of complications and so do not improve stroke prognosis [34–37]. Nutritional support therapy is an important intervention in the treatment of acute severe stroke. To account for treatment and provision of adequate nutrition for recovery in the later stages, most studies have adopted early EN maintenance therapy [38]. Researchers have also found that EN is suitable in patients with any consciousness disorders [39, 40]. However, Xu found that EN can cause a variety of gastrointestinal adverse reactions [41]. Probiotics can reduce complication rates and inhibit the growth of harmful bacteria in the intestine [42]. Using the principle of biological antagonism to adjust the balance of intestinal flora is also in line with modern medical treatment concepts.

However, the relationship between probiotics and stroke is more complex. Huang found that changes in intestinal flora can affect ischemic brain injury symptoms in mice [43]. Winek pretreated mouse stroke models with antibiotics and found that mice with complex gut microbiota had higher survival rates [44]. This suggests that microbiota imbalance may be a factor underlying the onset of stroke. Ritzel found that the incidence of intestinal dysbiosis in elderly patients after stroke is increasing [45]. Liao found an increase in pathogenic bacteria and a decrease in probiotics in the intestinal flora of patients with ischemic stroke [46]. The latest research has shown that gastrointestinal flora imbalance can affect stroke occurrence through a bottom-up signaling axis [47–49]. Thus, there may be a relationship between intestinal inflammation and immune response [50–52]. Probiotics and their metabolites, such as short-chain fatty acids, can significantly improve systemic inflammatory response syndrome in severely ill patients [53]. Also, the gut microbiota might be a target for stroke treatment [48], but this has yet to be supported by convincing evidence.

Meta-analysis is a statistical method that combines the results of several studies into a quantitative indicator. The combination of data from multiple studies can increase the sample size and improve a test's reliability. In this meta-analysis, we combined 23 RCTs of probiotics combined with EN in the treatment of stroke. Our findings showed that probiotics combined with EN did not reduce NIHSS scores (*P* > 0.05) but did reduce the duration of hospital stays and bedrest periods (*P* < 0.05). This suggests that probiotics combined with EN has a positive effect on stroke. Furthermore, probiotics combined with EN also improved patients' nutritional status by increasing their HB, ALB, TP, and PA content (*P* < 0.05), which is crucial to recovery. In terms of mitigating adverse reactions, our results indicate that the effect of probiotics combined with EN is significant; it relieves intestinal stress and reduces the occurrence of adverse reactions such as esophageal reflux, bloating, constipation, diarrhea, gastric retention, and gastrointestinal bleeding (*P* < 0.05). In terms of reducing stroke complications, we found that probiotics combined with EN reduced the incidence of lung infections, gastrointestinal infections, and urinary tract infections (*P* < 0.05). It also reduced the fatality intestinal flora imbalance rates (*P* < 0.05). These findings indicate that the combination of probiotics and EN has significant effects on both nutritional support and intestinal inflammation reduction.

In terms of improving inflammation, we found that probiotics combined with EN reduced hs-CRP and PCT, but this difference was not significant (*P* > 0.05). However, in reducing TNF-*α*, IL-6, and IL-10, the difference was significant (*P* < 0.05). TNF-*α* and IL-6 are the same type of inflammatory factor. When there is high permeability in the intestine, the intestinal microcirculation is destroyed, especially in the immature intestine. At this time, the intestinal artery is attacked by oxidative stress, and the vascular endothelial barrier is destroyed, which causes an abnormal acute microcirculation and an abnormality of the intestinal machinery barrier [54]. As an acute-phase reactive protein, CRP is secreted by hepatocytes after stimulation by inflammatory cells [55]. Under normal conditions, CRP content is very low, but it rises sharply when there is an acute inflammatory response caused by infection. PCT is a calcitonin precursor. Stimulation by inflammatory factors causes abundant secretion of PCT from the muscle, liver, and kidney. These inflammatory factors are negatively correlated with the prognosis of patients with stroke. Probiotics combined with EN is used to improve the imbalance of intestinal flora and intestinal local immunity [56]. Also, neuritis and cognitive dysfunction caused by endotoxins can be improved by probiotics [57]. These findings suggest that inflammatory responses can be reduced by probiotics combined with EN. Thus, the different results concerning inflammatory indicators are mainly produced by the small sample.

## 5. Limitations

The present systematic review has some limitations that should be noted. First, the methodological quality of the RCTs included was generally poor, and only 11 included studies [10, 13, 19, 21, 23, 26, 27, 29, 30] mentioned specific randomizing methods. No allocation concealment method or blinding method was mentioned for any of the RCTs, nor was it clear whether there were other biases. Second, the sample size of all the included studies was small, with a final total of only 1,816 patients. Third, this study primarily evaluated the effect of probiotics, but not all of the included studies listed the specific bacteria used. Therefore, it is impossible to evaluate each strain's independent influence on ischemic stroke. Fourth, the number of studies included in this meta-analysis was small. Finally, all of the included studies were published and reported positive results. Therefore, it was impossible to rule out the possibility of unpublished negative results.

## 6. Conclusion

In summary, additional rigorous randomized double-blind trials are needed to verify the safety and effectiveness of probiotics combined with EN in stroke treatment. However, this was a comprehensive meta-analysis of all published studies on the use of probiotics combined with EN in treating stroke that meet the standards. We objectively evaluated the clinical efficacy of probiotics combined with EN in treating stroke. Therefore, the results of the study still have significance for clinical guidelines.

## Figures and Tables

**Figure 1:** Document retrieval flowchart.

**Figure 2:** Funnel plots of publication bias analysis results.

**Table 1:** Basic information on the included literature.

Study	Disease	Course of treatment	Treatment group			Control group		
			Treatment	Male/female	Age	Treatment	Male/female	Age
Bai et al. [11]	IS + HS	1 w	PLBP + ENS	—	—	ENS	—	—
Ban et al. [12]	IS + HS	14 w	BLTLBT + ENS	25/10	65.8 ± 10.5	ENS	26/9	66.5 ± 8.3
Chen [13]	IS + HS	14d	BLTLBT + F	—	—	F	—	—
Chen et al. [14]	IS	14 d	PLBP + S	23/12	70.69 ± 11.68	S	19/15	71.37 ± 12.56
Dong [15]	IS + HS	14 d	PLBP + ENS	—	—	ENS	—	—
Feng [16]	IS	14 d	PLBP + FD	27/13	58.55 ± 8.67	FD	25/15	54.78 ± 7.74
Gao [17]	IS + HS	2 w	PLBP + ENS	21/19	58.2 ± 2.1	ENS	15/25	51.1 ± 2.3
Geng et al. [18]	IS	15 d	PP + ENS	33/24	65.8 ± 2.7	ENS	30/27	66.4 ± 22.4
He et al. [19, 20]	IS	1 m	PLBP + ENS	36/24	70.97 ± 10.86	ENS	16/14	69.21 ± 1 2.08
Huang and Yuan [20]	IS	21 d	BLTLBT + ENS	16/19	54.98 ± 5.10	ENS	15/20	55.21 ± 5.12
Jin [21]	IS	4 w	BTVEC + ENS	—	—	ENS	—	—
Jin et al. [22]	IS + HS	7–14 d	BLTLBT + ENS	13/15	62.18 ± 11.12	ENS	17/11	62.07 ± 10.94
Liang et al. [23]	HS	60 d	PLBP + FD	—	60.19 ± 18.65	FD	—	62.13 ± 13.97
Li et al. [24]	IS + HS	2 w	BQVT + ENS	29/11	—	ENS	28/12	—
Li [25]	HS	21 d	LCC + F	13/10	60.9 ± 8.7	F	14/8	59.5 ± 8.9
Li et al. [26]	HS	2 w	BLTLBT + ENE	24/19	60.90 ± 8.60	ENE	27/16	61.66 ± 10.64
Ma [27]	HS	20 d	BQVT + ENS	25/22	52 ± 6	ENS	26/20	52 ± 6
Pei [28]	IS + HS	4 w	PLBP + ENS	32/28	64 ± 10	ENS	35/25	62 ± 11
Yang [29]	IS + HS	7 w	PLBP + ENS	15/15	59.89 ± 3.46	ENS	17/13	60.23 ± 4.56
Yuan [30]	HS	2 w	BTVEC + HP	28/12	58.4 ± 9.3	HP	27/13	59.1 ± 8.8
Zhang [31]	IS	14 d	PLBP + EP	30/40	64.21 ± 9.27	EP	32/38	63.49 ± 10.64
Zhang et al. [32]	HS	21 d	LCC + F	13/10	60.9 ± 8.7	F	14/8	59.5 ± 8.9
Zhang [33]	IS + HS	8 w	LCBC	—	—	—	—	—

IS: ischemic stroke; HS: hemorrhagic stroke; m: month; w: week; d: day; PLBP: probiotic live bacteria preparation; BLTLBT: bifidobacterium lactobacillus triple live bacteria tablets; BTVEC: bifidobacterium triple viable enteric-coated capsules; PP: probiotic pellets; BQVT: bifidobacterium quadruple viable tablets; LCC: Livzon Changle capsules; LCBC: live clostridium butyricum capsules; EN: enteral nutrients; ST: life support treatment; F: fresubin; S: supportan; FD: fresubin diabetic; EP: ensure powder; HP: homogenate preparation; ENS: enteral nutrient solution or suspension; ENE: enteral nutrient emulsion.

**Table 2:** Quality evaluation results of the 21 included RCTs.

Study	Random sequence generation	Allocation hiding	Blind researchers and subjects	Blind evaluation of research results	Integrity of result data	Optional reporting of research results	Other biases
Bai et al.[11]	L	U	U	U	H	L	U
Ban et al. [12]	L	U	U	U	L	L	U
Chen et al. [13]	L	U	U	U	H	L	U
Chen et al. [14]	L	U	U	U	L	L	U
Dong [15]	U	U	U	U	H	L	U
Feng [16]	U	U	U	U	L	L	U
Gao [17]	U	U	U	U	L	L	U
Geng et al. [18]	U	U	U	U	L	L	U
He [19],	U	U	U	U	L	L	U
Huang and Yuan [20]	L	U	U	U	L	L	U
Jin et al. [22]	L	U	U	U	L	L	U
Liang et al. [23]	U	U	U	U	H	L	U
Li et al. [24]	L	U	U	U	H	L	U
Li [25]	U	U	U	U	H	L	U
Li et al. [26]	U	U	U	U	L	L	U
Ma [27]	L	U	U	U	L	L	U
Pei [28]	L	U	U	U	L	L	U
Yuan [30]	L	U	U	U	L	L	U
Zhang et al. [31]	L	U	U	U	L	L	U
Zhang et al. [32]	U	U	U	U	L	L	U
Zhang [33]	U	U	U	U	H	L	U

L: low risk; U: unknown risk; H: high risk.

**Table 3:** Quality evaluation results of the 2 included CCTs.

Study	Case definition adequacy	Case representativeness	Control selection	Definition of controls	Comparability of cases and controls	Exposure ascertainment	Uses the same method to determine case and control exposure factors	Nonresponse rate	Total
Jin [21]	★			★	★★		★	★	6
Yang [29]	★			★	★★		★	★	6

**Table 4:** Meta-analysis for continuous variables.

Effect index	Detail index	Studies included	Heterogeneity test	Model	MD (95% CI)
Effect on stroke	NIHSS score	2 [20, 31]	*I* ^*2*^ = 93%, *P*=0.0001	Random effects model	−1.11 (−7.92, 5.70), *P*=0.75
	Hospital stay duration	5 [17, 21, 23, 24, 29]	*I* ^*2*^ = 81%, *P*=0.0003	Random effects model	−8.94 (−11.39, −6.50), *P* < 0.00001
	Bedrest duration	3 [17, 24, 29]	*I* ^*2*^ = 0%, *P*=0.095	Fixed effects model	−10.34 (−11.30, −9.39), *P* < 0.00001

Blood nutrition indicators	HB	7 [12, 16, 21, 25, 26, 30, 31]	*I* ^*2*^ = 51%, *P*=0.06	Fixed effects model	8.36 (6.34, 10.38), *P* < 0.00001
	ALB	9 [12, 16, 21, 23, 25, 27, 30, 31]	*I* ^*2*^ = 54%, *P*=0.03	Random effects model	2.91 (2.45, 3.37), *P* < 0.00001
	TP	6 [16, 21, 25, 27, 31]	*I* ^*2*^ = 82%, *P* < 0.0001	Random effects model	4.90 (2.43, 7.38), *P* < 0.00001
	PA	4 [12, 16, 27, 31]	*I* ^*2*^ = 74%, *P*=0.01	Random effects model	15.50 (9.2, 21.79), *P* < 0.00001

Inflammation indicators	TNF-*α*	3 [14, 21, 26]	*I* ^*2*^ = 78%, *P*=0.01	Random effects model	−3.22 (−5.61, −0.82), *P* < 0.00001
	IL-6	2 [21, 26]	*I* ^*2*^ = 0%, *P*=0.40	Fixed effects model	−16.40 (−21.97, −10.83), *P* < 0.00001
	IL-10	2 [14, 23]	*I* ^*2*^ = 0%, *P*=0.50	Fixed effects model	−6.63 (−12.55, −0.70), *P* = 0.03
	hs-CRP	2 [14, 23]	*I* ^*2*^ = 0%, *P*=0.66	Fixed effects model	−2.82 (−10.10, 4.47), *P*=0.45
	PCT	2 [14, 23]	*I* ^*2*^ = 0%, *P*=0.53	Fixed effects model	−0.35 (−2.58, 1.89), *P*=0.76

**Table 5:** Binary variable meta-analysis results.

Effect index	Detail index	Study	Heterogeneity test	Model	RR (95% CI)
Adverse reactions	Vomiting	3 [16, 22, 27]	*I* ^*2*^ = 0%, *P*=0.90	Fixed effects model	0.83 (0.46, 1.51), *P*=0.55
	Stress ulcer	2 [22, 30]	*I* ^*2*^ = 14%, *P*=0.28	Fixed effects model	0.47 (0.22, 1.02), *P*=0.06
	Esophageal reflux	8 [11, 13, 16, 17, 22, 28, 29, 31]	*I* ^*2*^ = 29%, *P*=0.19	Fixed effects model	0.43 (0.25, 0.74), *P*=0.002
	Bloating	10 [11, 13, 17, 22, 27, 29, 31, 33]	*I* ^*2*^ = 0%, *P*=0.45	Fixed effects model	0.39 (0.26, 0.58), *P* < 0.00001
	Constipation	12 [11, 13, 16, 19, 23, 27, 29, 33]	*I* ^*2*^ = 0%, *P*=0.76	Fixed effects model	0.31 (0.21, 0.45), *P* < 0.00001
	Diarrhea	14 [11, 13, 16, 19, 22, 23, 27, 29, 31]	*I* ^*2*^ = 0%, *P*=0.93	Fixed effects model	0.22 (0.14, 0.34), *P* < 0.00001
	Gastric retention	4 [11, 13, 27–29]	*I* ^*2*^ = 0%, *P*=0.84	Fixed effects model	0.34 (0.19, 0.60), *P*=0.0002
	Gastrointestinal bleeding	10 [13, 15, 17, 19, 25, 26, 28, 29, 31]	*I* ^*2*^ = 0%, *P*=0.93	Fixed effects model	0.39 (0.28, 0.54), *P* < 0.00001

Complication rate	Lung infection	12 [11, 13, 15, 17, 25, 26, 28–32]	*I* ^*2*^ = 65%, *P*=0.0009	Random effects model	0.44 (0.27, 0.72), *P*=0.001
	Gastrointestinal infection	4 [11, 13, 17, 29]	*I* ^*2*^ = 0%, *P*=0.96	Fixed effects model	0.40 (0.23, 0.68), *P*=0.0008
	Urinary tract infection	6 [11, 13, 15, 17, 28, 29]	*I* ^*2*^ = 0%, *P*=0.93	Fixed effects model	0.27 (0.15, 0.49), *P* < 0.0001

Poor prognostic indicators	Mortality rate	4 [16, 17, 22, 29]	*I* ^*2*^ = 0%, *P*=0.44	Fixed effects model	0.45 (0.22, 0.93), *P*=0.03
	Bacterial imbalance rate	6 [11, 15, 25, 26, 28, 32]	*I* ^*2*^ = 0%, *P*=0.79	Fixed effects model	0.32 (0.21, 0.48), *P* < 0.0001

## Data Availability

Requests for additional data may be granted upon reasonable request by contacting the first author (Da-yuan Zhong, 13751728424@163.com) and the corresponding author (Yi-hui Deng, 644138330@qq.com).
